The article "lncRNA RP11-838N2.3 Promoted Cisplatin Resistance in Lung Adenocarcinoma" was published in 2020. Journal: Biomed Res Int.

# lncRNA RP11-838N2.3 Promoted Cisplatin Resistance in Lung Adenocarcinoma

**DOI:** 10.1155/2020/2806042

**Published:** 2020-06-14

**Authors:** Jie Chen, Feng Jiang, Lijuan Hu, Fan Zhang, Junjun Wang, Kate Huang, Yumin Wang

**Affiliations:** ^1^Department of Intensive Care Unit, The First Affiliated Hospital of Wenzhou Medical University, Wenzhou, China; ^2^Department of Laboratory Medicine, The First Affiliated Hospital of Wenzhou Medical University, Wenzhou, China; ^3^Department of Pathology, The First Affiliated Hospital of Wenzhou Medical University, Wenzhou, China

## Abstract

The mechanism of RP11-838N2.3 promoting cisplatin resistance in lung adenocarcinoma (LAD) was unclear. The RP11-838N2.3 expression level in cells and LAD tissues was detected by qPCR. We constructed lentivirus-mediated GV303 overexpression and GV248 shRNA vector targeting RP11-838N2.3, then infected A549 and A549/DDP cell and furtherly analyzed cell biology. High-throughput gene chip analysis showed that RP11-838N2.3 was significantly upregulated in A549/DDP (change fold = 66.056595). The qPCR results showed that the expression level of RP11-838N2.3 in A549/DDP cell was significantly higher than that in A549 cells (*P* < 0.05), and the expression level of RP11-838N2.3 in LAD tissues was also significantly higher than that in adjacent tissues (*P* < 0.05). The expression level of RP11-838N2.3 in cisplatin-insensitive LAD tissues was also significantly higher than that in cisplatin-sensitive LAD tissues (*P* < 0.05). Survival analysis showed that OS (overall survival) and DFS (progression-free survival) of high RP11-838N2.3 expression in the cisplatin-sensitive or cisplatin-insensitive LAD group were lower (*P* < 0.001 and *P* < 0.001) than those of low RP11-838N2.3 expression in the cisplatin-sensitive or cisplatin-insensitive LAD group. CCK8 showed that the OD450 value of RP11-838N2.3 overexpression increased significantly at 24 h, 48 h, and 72 h after transfection, while the knockdown of RP11-838N2.3 caused OD450 value at 24 h, 48 h, and 72 h after transfection significantly reduced, under the action of cisplatin that had the same trend (*P* < 0.05). The cell migration showed that the RP11-838N2.3 overexpression increased significantly migration activity and RP11-838N2.3 knockdown inhibited migration activity at 24 h, 48 h, and 72 h after transfection. The same trend was also observed under the action of cisplatin (*P* < 0.05). The cell invasion showed that the invasion rate of RP11-838N2.3 overexpression increased significantly, while the invasion rate of RP11-838N2.3 knockdown decreased significantly, and the same trend was observed under the action of cisplatin (*P* < 0.05). Apoptosis results showed that the apoptosis rate of RP11-838N2.3 overexpressed cells decreased significantly and the apoptosis rate of RP11-838N2.3 knockdown cells increased significantly, and the same trend was also observed under the action of cisplatin (*P* < 0.05). However, the results of cell cycle showed that there was no significant difference in the proportion of cells in each phase of the cell cycle after RP11-838N2.3 overexpression or knockdown (*P* > 0.05).RP11-838N2.3 was significantly upregulated in cisplatin-resistant cell and tissues of LAD. RP11-838N2.3 could enhance the proliferation, migration, and invasion and inhibit apoptosis of LAD cisplatin-resistant cell. So RP11-838N2.3 could enhance the cisplatin resistance of LAD cells and was a resistant lncRNA molecule.

The article "lncRNA RP11-838N2.3 Promoted Cisplatin Resistance in Lung Adenocarcinoma" was published in 2020. Journal: Biomed Res Int.

## 1. Introduction

Globally, the highest rate of incidence and mortality among all cancers is lung cancer. Lung adenocarcinoma (LAD), accounting for 40% of lung cancer, is one of the most common types of NSCLC. Though targeted and immunological drugs are constantly appearing, cisplatin-based combination chemistry played a key role in its comprehensive treatment program [1]. With the wide application of cisplatin, it will inevitably cause tumor cells to develop resistance to it, so that the chemotherapy effect is evidently reduced [2]. Studies had shown that in the early stage of chemotherapy, 70-80% patients could temporarily relieve lung cancer; however, long-term application would produce resistance to cisplatin, resulting in a recurrence rate of more than 60%, while drug resistance of recurrent lung cancer was clearly put up, with chemotherapy drug remission rate lower than 30% [3]; the current chemotherapy rate was only 30-40%, and the five-year survival rate was less than 15% in patients with advanced LAD [4]. According to the American Cancer Society survey, more than 90% of cancer patients' deaths were related to tumor drug resistance to varying degrees. Once cancer cells were resistant to cisplatin, they would be resistant to doxorubicin, vinblastine, fluorouracil, mitomycin, etc. Many first-line chemotherapeutic drugs form multidrug resistance, which was particularly harmful [5]. Therefore, seeking out specific molecular targets and biomarkers relative to cisplatin resistance in LAD and further reversing its cisplatin resistance would be of great significance for improving the prognosis of patients with LAD.

In recent years, studies at home and abroad have shown that cisplatin is a cell cycle nonspecific cytotoxic drug, which plays a role mainly by inhibiting DNA synthesis of tumor cells [6] and inducing apoptosis [7]. The mechanism of cisplatin resistance is extremely complex. It is a complex event involving multiple genes involved in multiple proteins and several pathways. It is currently believed to be achieved mainly through some mechanisms [6, 7, 8, 9, 10], However, it is regrettable that the mechanism of cisplatin resistance has not yet been elucidated, despite the genomics and proteomics progress in the past.

The article "lncRNA RP11-838N2.3 Promoted Cisplatin Resistance in Lung Adenocarcinoma" was published in 2020. Journal: Biomed Res Int.

Studies had shown that lncRNAs are involved in the cisplatin resistance mechanism of tumors including lung cancer [11, 12, 13], which provided an important opportunity to clarify the cisplatin resistance mechanism of tumor cells and to find ways to reverse cisplatin resistance. At present, research on 1ncRNAs in cisplatin resistance in lung cancer was still in its infancy, and some lncRNA molecules related to cisplatin resistance in lung cancer had been screened and identified, including H19 [12], XIST [14], SFTA1P [15], CCAT1 [16], and MALAT1 [17]. However, lncRNAs related to cisplatin resistance in lung cancer needed to be further explored for its mechanism of action.

We had previously used high-throughput lncRNA chip technology to compare LAD cisplatin-resistant A549/DDP cell with cisplatin-sensitive A549 cell to obtain differential lncRNA panel of cisplatin-resistant LAD. Expression profiles were screened and preliminarily identified several lncRNA molecules closely related to cisplatin resistance in LAD. We initially identified multiple lncRNA candidate genes of interest and verified them by qPCR. We found multiple lncRNA expressions and chips were consistent, indicating that the lncRNAs were involved in the process of cisplatin resistance in LAD, which was consistent with related reports [12, 14, 15, 16, 17]. Among them, we found that the lncRNA RP11-838N2.3 (also called LINC01895) were overexpressed in A549/DDP by gene chip and qPCR. The gene was located at 18p11.31 and the length of the RNA sequence is 404 bp. At present, no related literature had been reported about the lncRNA molecule. Therefore, we speculated that RP11-838N2.3 might be a new lncRNA closely related to and resistant to LAD cisplatin.

However, this mechanism of RP11-838N2.3 was not well understood in LAD with resistance to cisplatin. In this study, we overexpressed and knocked down RP11-838N2.3 basing on lentivirus technology and unveiled this mechanism.

## 2. Materials and Methods

### 2.1. Cell Culture

A549 and A549/DDP cells were added with an appropriate amount of RPMI1640 medium containing 10% calf serum, gently pipetted into a single cell suspension with a pipette, and the cell suspension was transferred to a cell culture flask with a pipette and placed at 37°C (5% CO_2_). A549/DDP was added to 2 *μ*g/ml cisplatin to maintain drug resistance. The cell growth state was observed to be good, and the cell passage was performed at a density of 70% to 90%.

The article "lncRNA RP11-838N2.3 Promoted Cisplatin Resistance in Lung Adenocarcinoma" was published in 2020. Journal: Biomed Res Int.

### 2.2. Human LAD Tissue Specimens

From August 2013 to August 2014, there were 57 patients with LAD samples and corresponding adjacent tissue samples were collected from patients at the first Affiliated Hospital of Wenzhou Medical University including 28 men and 29 women. Tissue types included 11 cases with low differentiation, 7 cases with low differentiation, 17 cases with moderate differentiation, 9 cases with high differentiation, and 13 cases with high differentiation. All were confirmed by histopathology as adenocarcinoma. Immediately after resection, LAD and matched adjacent tissue samples were frozen in liquid nitrogen. The study was approved by the Institutional Ethics Review Committee of the First Affiliated Hospital of Wenzhou Medical University.

### 2.3. Cisplatin-Treated LAD Samples

Human LAD tissue specimens were collected in the First Affiliated Hospital of Wenzhou Medical University from 2010 to 2015. The specimens were obtained by lung puncture biopsy, surgical resection, and lymph node metastasis biopsy and were strictly identified by the Department of Pathology. All tissue specimens must meet the following conditions: primary LAD patients and clinical stage IIIB~IV. The first-line chemotherapy regimen was cisplatin 25 mg/m^2^, on 1-3 days, combined with gemcitabine 1000 mg/m^2^ or paclitaxel 80 mg/m^2^, on 1 and 8 days. The 21 days was a cycle, and each patient was treated for 3-4 cycles. According to CT, MRI, and other medical imaging examinations, serum tumor markers, and RECIST standard, they were divided into the “cisplatin-sensitive group” (complete remission+partial remission) and “cisplatin-insensitive group” (progress). There were 25 sensitive specimens and 32 insensitive specimens. Tissue specimens are stored in liquid nitrogen before use. The study was approved by the Institutional Ethics Review Committee of the First Affiliated Hospital of Wenzhou Medical University.

### 2.4. Constructed Lentivirus-Mediated Overexpression and shRNA Vector

The overexpression vector targeting RP11-838N2.3 (OE) as well as a negative control (OE-NC) (Genechem, Shanghai, China) transfected A549 cell. According to experimental requirements, these groups were divided into A549 OE-NC, A549 OE-NC+2 *μ*g/ml cisplatin, A549 OE, and A549 OE+2 *μ*g/ml cisplatin. A549/DDP cell was transfected shRNA vector targeting RP11-838N2.3 (shRNA) as well as a negative control (shRNA NC) (Genechem, Shanghai, China); shRNA included four sequences—shRNA-1: 5′-TTCCTTCAGCCTCCAGGAATA-3′, shRNA-2: 5′-CTCTTTAGGGAC AGAGAGGAA-3′, shRNA-3: 5′-ATGGCAGGAGCAAGTGGTTAT-3′, and shRNA-NC: 5′-TTCTCCGAACGTGTCACGT-3′. The optimal interfering sequence was screened by three shRNA sequence experiments as the subsequent experimental group. These groups were divided into A549/DDP shRNA-NC, A549/DDP shRNA-NC+2 *μ*g/ml cisplatin, A549/DDP shRNA, and A549/DDP shRNA+2 *μ*g/ml cisplatin. Transfection was performed with adding 2 × 10^5^ cells into a six-well plate, and after 24 h, the medium was aspirated and incubated with transfection complex abiding by the manufacturer's protocol and MOI value (MOI = 5). These cells were infected by lentivirus for 72 h and treated with 2 *μ*g/ml puromycin; further, qPCR detected the overexpression or shRNA efficiency.

The article "lncRNA RP11-838N2.3 Promoted Cisplatin Resistance in Lung Adenocarcinoma" was published in 2020. Journal: Biomed Res Int.

### 2.5. Quantitative PCR

Total RNAs of cells and tissues were obtained with TRizol reagent (Invitrogen). Total RNA was reverse-transcribed into cDNA using an RT Reagent Kit (Shanghai Takara, China), complying with the manufacturer's instructions. RP11-838N2.3 level expression was measured by qPCR in ABI 7500 instrument: RP11-838N2.3 for upstream primer: 5′-CAGGACTCAGAGCCTTTCCG-3′, downstream primer: 5′-GCCCTTGCCTGGATTACCAT-3′; *β*-actin for upstream primer: 5′-CATGTACGTTGCTATCCAGGC-3′, downstream primer: 5′-CTCCTTAATGTC ACGCACGAT-3′. 20 *μ*l PCR reaction volume included 6 *μ*l double-distilled water, 10 *μ*l SYBR Premix mixture (2×), 1 *μ*l PCR forward primer (10 mM), 1 *μ*l PCR reverse primer (10 mM), and 2 *μ*l cDNA template. The qPCR reaction program included a denaturation step of 10 min at 95°C, 40 cycles (5 s at 95°C, 30s at 60°C), and a final extension step of 5 min at 72°C. All samples were normalized to *β*-actin. The relative target gene concentration was calculated using the median triplicate (ΔCt = Ct median target gene − Ct median *β*‐actin), and 2^-*ΔΔ*Ct^ in expression was calculated.

### 2.6. Cell Scratch Test to Detect Cell Migration Ability

According to the principle of drawing 3 horizontal lines in each well, draw a horizontal line mark on the back of the 6-well plate with a marker pen, and add about 5 × 10^5^/well of cell lines and make 3 holes each. After incubation at 37°C, with 5% CO_2_, cells were spread on the bottom of the plate; we used 10 *μ*l pipette tips to make cell scratches perpendicular to the well plate and tried to ensure that the width of each scratch was consistent. We washed the cells 3 times with PBS, add serum-free medium, took pictures, and recorded it. The culture plate was placed in an incubator for cultivation, and pictures were taken.

### 2.7. Cell Migration Assays

It was carried out in 24 well plates, and the insertion well is 8 *μ*m (Milipole Company of the United States). 2 × 10^4^ cells were added to the cavity on the orifice plate. Methanol was fixed; 0.1% (w/w) crystal violet staining, 33% acetic acid bleaching, and 570 nm absorbance were measured.

The article "lncRNA RP11-838N2.3 Promoted Cisplatin Resistance in Lung Adenocarcinoma" was published in 2020. Journal: Biomed Res Int.

### 2.8. Cell Viability Assay

According to the manufacturer's plan, the cell count kit-8 (Corning, UAS) was used to evaluate it. 3000 cells and a complete medium containing 10% fetal bovine serum were added to the 96-well plate. On the second day, A549/DDP or A549 cells were incubated with CCK8 for 1 h, and the absorbance of 450 nm was measured by (TECAN) at 0 h, 24 h, 48 h, and 72 h. The experiment was carried out in tetraploid cells.

### 2.9. Flow Cytometry to Detect Apoptotic Rate

5 × 10^5^ cells were collected and washed with PBS twice. Suspension cells were added with 500 *μ*l binding buffer, and 1 *μ*l Annexin V-PE was added to the mixture at room temperature. After adding 5 *μ*l 7-AAD solution and shaking 15 min at room temperature, the cells were observed and detected by a fluorescence microscope or flow cytometry.

### 2.10. Cell Cycle Assay

The cells of each experimental group were collected by centrifugation and fixed with 70% ethanol at 4°C for a period. The cells were then suspended in 400 *μ*l PBS containing 2 mg/ml ribonuclease and incubated for 30 min at 37°C. Add 400 *μ*l propidium iodide (0.1 mg/ml) in 10 min. The content of DNA was detected by a cell cycle analyzer (Cyclinics FS500, Beckman), and the results were statistically analyzed by multicycle software.

### 2.11. Statistical Methods

The one-way ANOVA or Kruskal-Wallis test for the normal distribution was used to test the differences among three and more groups, and Student's *t*-test or Mann-Whitney *U* test was performed for the comparison between the two groups. A chi-square test was performed for survival analysis. *P* < 0.05 was statistically significant.

## 3. Results

### 3.1. QPCR Preliminary Verification of RP11-838N2.3 and Survival Analysis in LAD

Gene chip results showed that lncRNA RP11-838N2.3 expression was significantly upregulated in A549/DDP cell (change fold = 66.056595). QPCR results showed that the expression level of RP11-838N2.3 in cisplatin-resistant A549/DDP cells was plainly higher than that in cisplatin-sensitive A549 cells (Mann-Whitney *U* test = 0.000, *P* ≤ 0.001). The RP11-838N2.3 expression level of LAD was also clearly higher than that of adjacent tissues (Mann-Whitney *U* test = 12.32, *P* = 0.001). Further research showed that the RP11-838N2.3 level of LAD with lymph node metastasis was significantly higher than that of the no lymph node metastasis group (Mann-Whitney *U* test = 3.213, *P* = 0.009). RP11-838N2.3 expression levels among sex (Mann-Whitney *U* test = 234.00, *P* = 0.453), clinical stages (Kruskal-Wallis *U* test = 10.124, *P* = 0.414), histology differentiation (Kruskal-Wallis *U* test = 11.456, *P* = 0.321), and smoking (Mann-Whitney *U* test = 267.00, *P* = 0.627) were not different (shown in Table 1).

The article "lncRNA RP11-838N2.3 Promoted Cisplatin Resistance in Lung Adenocarcinoma" was published in 2020. Journal: Biomed Res Int.

The result suggested that the expression level of RP11-838N2.3 in the cisplatin-insensitive LAD group was also significantly higher than that in the cisplatin-sensitive LAD group (Mann-Whitney *U* test = 0.000, *P* < 0.0001), as shown in Figure 1. In order to ensure the comparability of the tissue sample data, our findings showed that there were no differences of clinical characteristics between the cisplatin-sensitive group and the cisplatin-insensitive group, as shown in Table 2. Survival analysis showed that OS (overall survival) and DFS (progression-free survival) of high RP11-838N2.3 expression in the cisplatin-sensitive LAD group were lower (*P* < 0.001 and *P* < 0.001) than those of low RP11-838N2.3 expression in the cisplatin-sensitive LAD group; similarly, OS and DFS of high RP11-838N2.3 expression in the cisplatin-insensitive LAD group were lower (*P* < 0.001 and *P* < 0.001) than those of low RP11-838N2.3 expression in the cisplatin-insensitive LAD group, as shown in Figure 2.

### 3.2. Construction of Overexpression and shRNA Vector and Transfection Cells

A549/DDP cells were transfected with three groups of RP11-838N2.3 shRNA vectors. The shRNA-2 and shRNA-3 expression levels were plainly lower than the NC and shRNA-1group, and the differences were statistically significant (*P* < 0.001). Among them, the shRNA-2 group has the highest interference efficiency, as shown in Figure 3(a), indicating that the shRNA interference vector was successfully transfected. So the cells of the shRNA-2 group will be used for subsequent experiments. The expression level of RP11-838N2.3 in A549 cells transfected with the overexpression vector was plainly higher than that in the NC group (*P* < 0.01), indicating that the overexpression vector was successfully transfected, as shown in Figure 3(b).

### 3.3. Regulating Expression of RP11-838N2.3 Could Affect Proliferation Efficiency of A549 and A549/DDP Cells

Compared with that of 0 h, the OD450mn of 24 h (*P* < 0.001, *P* < 0.001, *P* < 0.001, and *P* < 0.001), 48 h (*P* < 0.001, *P* < 0.001, *P* < 0.001, and *P* < 0.001), 72 h (*P* < 0.001, *P* < 0.001, *P* < 0.001, *P* < 0.001, and *P* = 0.001) plainly increased. Compared with that of the A549 OE-NC group, the OD450mn of the A549 OE group increased significantly in 24 h (*F* = 0.406, *P* = 0.005), 48 h (*F* = 0.680, *P* = 0.001), and 72 h (*F* = 10.221, *P* = 0.04). Under the action of 2 *μ*g/ml cisplatin drug, RP11-838N2.3 overexpression still plainly promoted the proliferation of A549 cell. Compared with that of the A549 OE-NC+2 *μ*g/ml cisplatin group, the OD450mn of the A549 OE+2 *μ*g/ml cisplatin group in 24 h (*F* < 0.001, *P* = 0.004), 48 h (*F* = 11.270, *P* = 0.015), and 72 h (*F* = 6.486, *P* = 0.033) all increased significantly, as shown Figure 4. So RP11-838N2.3 overexpression plainly promotes the proliferation of A549 cells.

The article "lncRNA RP11-838N2.3 Promoted Cisplatin Resistance in Lung Adenocarcinoma" was published in 2020. Journal: Biomed Res Int.

Compared with that of 0 h, the OD450mn of 24 h (*P* < 0.001, *P* < 0.001, *P* < 0.001, and *P* < 0.001), 48 h (*P* < 0.001, *P* < 0.001, *P* < 0.001, and *P* < 0.001), and 72 h (*P* < 0.001, *P* < 0.001, *P* < 0.001, *P* < 0.001, and *P* = 0.001) significantly reduced. Compared with that of the A549/DDP shRNA-NC group, the OD450mn of the A549/DDP shRNA group in 24 h (*F* = 1.101, *P* = 0.002), 48 h (*F* = 0.525, *P* < 0.001), and 72 h (*F* = 0.889, *P* < 0.001) plainly reduced. Under the action of cisplatin drugs, RP11-838N2.3 knockdown can still obviously inhibit the proliferation of A549/DDP cells. Compared with that of the A549/DDP shRNA-NC+2 *μ*g/ml cisplatin group, the OD450mn of A549/DDP shRNA+2 *μ*g/ml cisplatin group in 24 h (*F* = 0.130, *P* = 0.001), 48 h (*F* = 1.482, *P* = 0.001), and 72 h (*F* = 0.006, *P* < 0.001) significantly reduced, as shown in Figure 5. Therefore, RP11-838N2.3 knockdown obviously inhibited the proliferation of A549/DDP cells.

### 3.4. Regulating RP11-838N2.3 Expression Could Affect Migration Ability of A549 and A549/DDP Cells

Compared with that of 0 h, the relative widths of 24 h (*P* < 0.001, *P* < 0.001, *P* < 0.001, and *P* < 0.001), 48 h (*P* < 0.001, *P* < 0.001, *P* < 0.001, and *P* < 0.001), and 72 h (*P* < 0.001, *P* < 0.001, *P* < 0.001, and *P* < 0.001) all decreased obviously, and the migration increased significantly. Compared with that of the A549 OE-NC group, the relative widths of the A549 OE group in 24 h (*F* = 0.407, *P* < 0.001), 48 h (*F* = 3.048, *P* < 0.001), and 72 h (*F* = 0.661, *P* < 0.001) decreased evidently, so the mobility increased significantly. The result hinted that RP11-838N2.3 overexpression evidently promoted the migration of A549 cells. Under the action of cisplatin drugs, RP11-838N2.3 overexpression still clearly promoted the migration of A549 cells. Compared with that of the A549 OE-NC+2 *μ*g/ml cisplatin group, the relative widths of the A549 OE+2 *μ*g/ml cisplatin group in 24 h (*F* = 1.140, *P* < 0.001), 48 h (*F* = 7.576, *P* < 0.001), and 72 h (*F* = 1.102, *P* < 0.001) decreased evidently and the mobility increased clearly, as shown in Figure 6.

Compared with that of 0 h, the relative widths of 24 h (*P* < 0.001, *P* < 0.001, *P* < 0.001, and *P* < 0.001), 48 h (*P* < 0.001, *P* < 0.001, *P* < 0.001, and *P* < 0.001), and 72 h (*P* < 0.001, *P* < 0.001, *P* < 0.001, and *P* = 0.001) decreased obviously and the mobility increased evidently. Compared with that of the A54/DDP shRNA-NC group, the relative widths of A549/DDP shRNA group in 24 h (*F* = 0.007, *P* < 0.001), 48 h (*F* = 0.914, *P* < 0.001), and 72 h (*F* = 0.007, *P* < 0.001) increased obviously, and the mobility decreased clearly. These results showed that RP11-838N2.3 knockdown obviously inhibited the migration of A549/DDP cells. Under the action of cisplatin drugs, RP11-838N2.3 gene knockdown can still clearly inhibit the migration of A549/DDP cells. Compared with that of the A549/DDP shRNA-NC+2 *μ*g/ml cisplatin group, the relative widths of A549/DDP shRNA+2 *μ*g/ml cisplatin group in 24 h (*F* = 2.129, *P* < 0.001), 48 h (*F* = 2.919, *P* < 0.001), and 72 h (*F* = 5.460, *P* < 0.001) increased clearly, and the mobility decreased obviously, as shown in Figure 7.

The article "lncRNA RP11-838N2.3 Promoted Cisplatin Resistance in Lung Adenocarcinoma" was published in 2020. Journal: Biomed Res Int.

### 3.5. Regulating RP11-838N2.3 Expression Affected Clear Invasion Ability of A549 and A549/DDP Cells

Compared with that of the A549 OE-NC group, the relative invasion rate of the A549 OE group increased significantly (*F* = 0.446, *P* < 0.001). Under the action of cisplatin drugs, RP11-838N2.3 gene overexpression still significantly promoted the proliferation of A549 cells. Compared with that of the A549 OE-NC+2 *μ*g/ml cisplatin group, the relative invasion rate of the A549 OE+2 *μ*g/ml cisplatin group increased obviously (*F* = 3.985, *P* < 0.001) as shown in Figure 8. So RP11-838N2.3 overexpression clearly promoted the invasion of A549 cells.

Compared with that of the A549/DDP shRNA-NC group, the relative invasion rate of the A549/DDP shRNA group was obviously reduced (*F* = 2.091, *P* < 0.001). Under the action of cisplatin drugs, RP11-838N2.3 gene knockdown can still distinctly inhibit the invasion of A549/DDP cells. Compared with that of the A549/DDP shRNA-NC+2 *μ*g/ml cisplatin group, the relative invasion rate of the A549/DDP shRNA+2 *μ*g/ml cisplatin group still decreased clearly (*F* = 0.248, *P* < 0.001) as shown in Figure 9. So RP11-838N2.3 knockdown distinctly inhibited the invasion of A549/DDP cells.

### 3.6. Regulating RP11-838N2.3 Expression Could Not Affect the Cell Cycle of A549 and A549/DDP Cells

Compared with those of the A549 OE-NC group, the cell ratios of the A549 OE group in the G0/G1 phase (*F* = 0.578,*P* = 0.051), S phase (*F* = 0.109,*P* = 0.397), and G2/M phase (*F* = 0.649,*P* = 0.992) were no significantly different. Under the action of cisplatin, compared with those in the A549 OE-NC+2 *μ*g/ml cisplatin group, the cell ratios A549 OE+2 *μ*g/ml cisplatin group in the G0/G1 phase (F =6.438, P =0.635), S phase (F =7.866, P =0.830), and G2/M phase (F =0.836, P =0.488) were not distinctly different, as shown in Figure 10. Compared with those in the A549/DDP shRNA-NC group, the cell ratios in the A549/DDP shRNA group in the G0/G1 phase (*F* = 1.012, *P* = 0.905), the S phase (*F* = 0.341, *P* = 0.221), and G2/M phase (*F* = 1.942, *P* = 0.110) were not evidently different. Under the action of cisplatin, compared with those in the A549/DDP shRNA-NC+2 *μ*g/ml cisplatin group, the cell ratios in the A549/DDP shRNA+2 *μ*g/ml cisplatin group in the G0/G1 phase (*F* = 0.958, *P* = 0.400), S phase (*F* = 11.701, *P* = 0.662), and G2/M phase (*F* = 8.507, *P* = 0.248) were not different. There were also no significant differences in the proportion of cells, as shown in Figure 11. So regulating RP11-838N2.3 expression could not affect the cell cycle of A549 and A549/DDP cells.

The article "lncRNA RP11-838N2.3 Promoted Cisplatin Resistance in Lung Adenocarcinoma" was published in 2020. Journal: Biomed Res Int.

### 3.7. Apoptosis of A549 and A549/DDP Cells Was Clearly Changed after Regulating RP11-838N2.3 Expression

Compared with that of the A549 OE-NC group, the apoptosis rate of the A549 OE group was evidently reduced (*F* = 10.304, *P* = 0.001). Under the action of cisplatin drugs, RP11-838N2.3 overexpression still significantly inhibited the apoptosis of A549. Compared with that of the A549 OE-NC+2 *μ*g/ml cisplatin group, the apoptosis rate of the A549 OE+2 *μ*g/ml cisplatin group also decreased clearly (*F* = 2.236, *P* < 0.001), as shown in Figure 12. So RP11-838N2.3 overexpression evidently inhibited the apoptosis of A549 cells.

Compared with that of the A549/DDP shRNA-NC group, the apoptosis rate of the A549/DDP shRNA group was evidently increased (*F* = 5.828, *P* < 0.001). Under the action of cisplatin drugs, RP11-838N2.3 knockdown can also evidently promote the apoptosis of A549/DDP cell. Compared with that of the A549/DDP shRNA-NC+2 *μ*g/ml cisplatin group, the apoptosis rate of the A549/DDP shRNA+2 *μ*g/ml cisplatin group was also evidently increased (*F* = 3.322, *P* < 0.001), as shown in Figure 13. So RP11-838N2.3 knockdown evidently promoted the apoptosis of A549/DDP cells.

## 4. Discussion

The mechanism of cisplatin resistance was extremely complex and involved multiple genes, multiple proteins and several pathways. It is currently believed to be achieved mainly through the following mechanisms [6, 7, 8, 9, 10]: (1) altering intracellular drug transport, such as ATP binding cassette protein; (2) reducing interference of drug ability with some mechanisms; (3) affecting DNA damage relative repairing gene, as breast cancer related gene 1 (BRCA1), excision repair cross-complementing gene (ERCC1), etc.; and (4) resulting genetic and epigenetic changes of the main signaling pathways.

The article "lncRNA RP11-838N2.3 Promoted Cisplatin Resistance in Lung Adenocarcinoma" was published in 2020. Journal: Biomed Res Int.

Many studies had confirmed that long noncoding RNA might be closely related to cisplatin resistance in LAD. Studies have shown that AK126698 regulates NSCLC cisplatin resistance by targeting the Frizzled-8 gene and partly through the Wnt signaling pathway [18]. MEG3 expression reduced A549/DDP by inducing activation of the mitochondrial apoptotic pathway p53 protein and Bcl-xl to cell cisplatin resistance [19]. NEAT1 increases the sensitivity of NSCLC to cisplatin by inhibiting hsa-mir-98-5p upregulating the expression of CTR1 induced by EGCG [20].

Our findings shown that the expression of RP11-838N2.3 in A549/DDP was evidently increased from high-throughput gene chip. The qPCR showed that the expression of RP11-838N2.3 in A549/DDP was evidently higher than that in A549. The expression level of RP11-838N2.3 of primary cultured cisplatin-insensitive LAD was also significantly higher than that of cisplatin-sensitive LAD. Our findings shown that there were no differences of clinical characteristics between the cisplatin-sensitive group and the cisplatin-insensitive group, so the tissue sample data were comparable. Survival analysis showed that OS (overall survival) and DFS (progression-free survival) of high RP11-838N2.3 expression in the cisplatin-sensitive or cisplatin-insensitive LAD group were lower (*P* < 0.001 and *P* < 0.001) than those of low RP11-838N2.3 expression in the cisplatin-sensitive or cisplatin-insensitive LAD group. The above results suggested that RP11-838N2.3 might be a drug resistance gene that could enhance cisplatin resistance in LAD.

In this study, RP11-838N2.3 overexpression vector and shRNA interference vector were successfully constructed through lentiviral vector technology, and the corresponding cells were transfected to obtain overexpressing A549 cell and knockdown A549/DDP cell. The results showed that RP11-838N2.3 overexpression enhanced proliferation, migration, and invasion capabilities of A549 cells and cell apoptosis was evidently inhibited. After RP11-838N2.3 knockdown, A549/DDP was evidently inhibited in their proliferation, migration, and invasion capabilities and apoptosis was evidently enhanced. The above results illustrated the role of RP11-838N2.3 in cisplatin resistance of LAD, suggesting the potential of RP11-838N2.3 as a gene therapy for LAD.

In summary, our study clearly identified that RP11-838N2.3 was evidently upregulated in A549/DDP, and cytological experiments confirmed that RP11-838N2.3 enhanced cell proliferation, migration, and invasion and inhibit apoptosis to enhance cisplatin resistance of LAD cells and provided a new therapeutic target for LAD treatment.

The article "lncRNA RP11-838N2.3 Promoted Cisplatin Resistance in Lung Adenocarcinoma" was published in 2020. Journal: Biomed Res Int.

## Figures and Tables

**Figure 1:** The expression level of RP11-838N2.3 in LAD tissues, adjacent tissues, and cells. (a) RP11-838N2.3 expression level in A549/DDP and A549 cell. (b) RP11-838N2.3 expression level in LAD and adjacent tissues. (c) The expression levels of lncRNA RP11-838N2.3 in cisplatin-sensitive LAD cells and cisplatin-insensitive LAD cells were primary cultured. QPCR results showed that the expression level of RP11-838N2.3 in cisplatin-resistant A549/DDP cell was plainly higher than that in cisplatin-sensitive A549 cell (Mann-Whitney *U* test = 0.000, *P* ≤ 0.001). The RP11-838N2.3 expression level of LAD was also clearly higher than that of adjacent tissues (Mann-Whitney *U* test = 12.32, *P* = 0.001). ^###^*P* < 0.001; ^∗∗^*P* < 0.01.

**Figure 2:** Survival analysis of the expression level of RP11-838N2.3 in LAD. (a) Survival analysis shown that OS (overall survival) of high RP11-838N2.3 expression in the cisplatin-sensitive LAD group was lower (*P* < 0.001) than that of low RP11-838N2.3 expression in the cisplatin-sensitive LAD group. (b) Survival analysis showed that DFS (progression-free survival) of high RP11-838N2.3 expression in the cisplatin-sensitive LAD group was lower (*P* < 0.001) than that of low RP11-838N2.3 expression in the cisplatin-sensitive LAD group. (c) OS of high RP11-838N2.3 expression in the cisplatin-insensitive LAD group was lower (*P* < 0.001) than that of low RP11-838N2.3 expression in the cisplatin-insensitive LAD group. (d) DFS of high RP11-838N2.3 expression in the cisplatin-insensitive LAD group was lower (*P* < 0.001) than that of low RP11-838N2.3 expression in the cisplatin-insensitive LAD group.

**Figure 3:** Construction of overexpression and shRNA vector and transfection cells. (a) A549/DDP cells were transfected with three groups of RP11-838N2.3 shRNA vectors. The shRNA-2 and shRNA-3 expression levels were plainly lower than the NC and shRNA-1 groups, and the differences were statistically significant (*P* < 0.001). Among them, the shRNA-2 group has the highest interference efficiency. (b) The expression level of RP11-838N2.3 in LAD cisplatin-sensitive A549 cells transfected with the overexpression vector was plainly higher than that in the NC group (*P* < 0.01). ^∗∗^*P* < 0.01; ^∗∗∗^*P* < 0.001.

**Figure 4:** Overexpression of RP11-838N2.3 could enhance proliferation efficiency of A549. (a) Compared with that of 0 h, the OD450mn of 24 h (*P* < 0.001, *P* < 0.001, *P* < 0.001, and *P* < 0.001), 48 h (*P* < 0.001, *P* < 0.001, *P* < 0.001, and *P* < 0.001), and 72 h (*P* < 0.001, *P* < 0.001, *P* < 0.001, *P* < 0.001, and *P* = 0.001) plainly increased. Compared with that of the A549 OE-NC group, the OD450mn of the A549 OE group increased significantly in 24 h (*F* = 0.406, *P* = 0.005), 48 h (*F* = 0.680, *P* = 0.001), and 72 h (*F* = 10.221, *P* = 0.04). (b) Under the action of 2 *μ*g/ml cisplatin drug, RP11-838N2.3 overexpression still plainly promoted the proliferation of A549 cells. Compared with that of the A549 OE-NC+2 *μ*g/ml cisplatin group, the OD450mn of A549 OE+2 *μ*g/ml cisplatin group in 24 h (*F* < 0.001, *P* = 0.004), 48 h (*F* = 11.270, *P* = 0.015), and 72 h (*F* = 6.486, *P* = 0.033) all increased significantly. ^∗^*P* < 0.05; ^∗∗^*P* < 0.01.

The article "lncRNA RP11-838N2.3 Promoted Cisplatin Resistance in Lung Adenocarcinoma" was published in 2020. Journal: Biomed Res Int.

**Figure 5:** Knockdown of RP11-838N2.3 could inhibit proliferation efficiency of A549/DDP. (a) Compared with that of 0 h, OD450mn of 24 h (*P* < 0.001, *P* < 0.001, *P* < 0.001, and *P* < 0.001), 48 h (*P* < 0.001, *P* < 0.001, *P* < 0.001, and *P* < 0.001), and 72 h (*P* < 0.001, *P* < 0.001, *P* < 0.001, *P* < 0.001, and *P* = 0.001) significantly reduced. Compared with the A549/DDP shRNA-NC group, the OD450mn of the A549/DDP shRNA group in 24 h (*F* = 1.101, *P* = 0.002), 48 h (*F* = 0.525, *P* < 0.001), and 72 h (*F* = 0.889, *P* < 0.001) plainly reduced. (b) Under the action of cisplatin drugs, RP11-838N2.3 gene knockdown can still obviously inhibit the proliferation of A549/DDP. Compared with the A549/DDP shRNA-NC+2 *μ*g/ml cisplatin group, the OD450mn of the A549/DDP shRNA+2 *μ*g/ml cisplatin group in 24 h (*F* = 0.130, *P* = 0.001), 48 h (*F* = 1.482, *P* = 0.001), and 72 h (*F* = 0.006, *P* < 0.001) significantly reduced. ^∗^*P* < 0.05; ^∗∗^*P* < 0.01.

**Figure 6:** Overexpression of RP11-838N2.3 could enhance migration ability of A549. (a) Compared with that of 0 h, the relative widths of 24 h (*P* < 0.001, *P* < 0.001, *P* < 0.001, and *P* < 0.001), 48 h (*P* < 0.001, *P* < 0.001, *P* < 0.001, and *P* < 0.001), and 72 h (*P* < 0.001, *P* < 0.001, *P* < 0.001, and *P* < 0.001) all decreased obviously, and the mobility increased significantly. Compared with the A549 OE-NC group, the relative widths of the A549 OE group in 24 h (*F* = 0.407, *P* < 0.001), 48 h (*F* = 3.048, *P* < 0.001), and 72 h (*F* = 0.661, *P* < 0.001) decreased evidently, and the mobility increased significantly. The result hinted that RP11-838N2.3 overexpression evidently promotes the migration of A549 cells. (b) Under the action of cisplatin drugs, RP11-838N2.3 overexpression still clearly promoted the migration of A549 cells. Compared with the that of the A549 OE-NC+2 *μ*g/ml cisplatin group, the relative widths of the A549 OE+2 *μ*g/ml cisplatin group in 24 h (*F* = 1.140, *P* < 0.001), 48 h (*F* = 7.576, *P* < 0.001), and 72 h (*F* = 1.102, *P* < 0.001) decreased evidently and the mobility increased clearly. ^∗∗∗^*P* < 0.01.

The article "lncRNA RP11-838N2.3 Promoted Cisplatin Resistance in Lung Adenocarcinoma" was published in 2020. Journal: Biomed Res Int.

**Figure 7:** Knockdown of RP11-838N2.3 could inhibit proliferation efficiency of A549/DDP. (a) Compared with that of 0 h, the relative widths of 24 h (*P* < 0.001, *P* < 0.001, *P* < 0.001, and *P* < 0.001), 48 h (*P* < 0.001, *P* < 0.001, *P* < 0.001, and *P* < 0.001), 72 h (*P* < 0.001, *P* < 0.001, *P* < 0.001, and *P* < 0.001) decreased obviously and the mobility increased evidently. Compared with that of the A54/DDP shRNA-NC group, the relative widths of the A549/DDP shRNA group in 24 h (*F* = 0.007, *P* < 0.001), 48 h (*F* = 0.914, *P* < 0.001), and 72 h (*F* = 0.007, *P* < 0.001) increased obviously, and the mobility decreased clearly. These results showed that RP11-838N2.3 knockdown obviously inhibited the migration of A549/DDP cells. (b) Under the action of cisplatin drugs, RP11-838N2.3 knockdown can still clearly inhibit the migration of A549/DDP cells. Compared with that of the A549/DDP shRNA-NC+2 *μ*g/ml cisplatin group, the relative widths of the A549/DDP shRNA+2 *μ*g/ml cisplatin group in 24 h (F =2.129, *P* < 0.001), 48 h (F =2.919, *P* < 0.001), and 72 h (F =5.460, P <0.001) increased clearly. ^∗∗∗^*P* < 0.01.

**Figure 8:** Overexpression of RP11-838N2.3 could enhance invasion ability of A549. (a) A549 OE-NC. (b) A549 OE. (c) A549 OE-NC+2 *μ*g/ml cisplatin. (d) A549 OE+2 *μ*g/ml cisplatin. (e) Compared with the A549 OE-NC group, the relative invasion rate of the A549 OE group increased significantly (*F* = 0.446, *P* < 0.001). Under the action of cisplatin drugs, RP11-838N2.3 gene overexpression still significantly promoted the proliferation of A549 cells. Compared with that of the A549 OE-NC+2 *μ*g/ml cisplatin group, the relative invasion rate of the A549 OE+2 *μ*g/ml cisplatin group increased obviously (*F* = 3.985, *P* < 0.001) as shown in Figure 7. So RP11-838N2.3 overexpression clearly promoted the invasion of strain A549 cells. ^∗∗∗^*P* < 0.01.

**Figure 9:** Knockdown of RP11-838N2.3 could inhibit invasion ability of A549/DDP (a) A549/DDP shRNA-NC. (b) A549/DDP shRNA. (c) A549/DDP shRNA-NC+2 *μ*g/ml cisplatin. (d) A549/DDP shRNA+2 *μ*g/ml cisplatin. (e) Compared with that of the A549/DDP shRNA-NC group, the relative invasion rate of the A549/DDP shRNA group was obviously reduced (*F* = 2.091, *P* < 0.001). Under the action of cisplatin drugs, RP11-838N2.3 gene knockdown can still distinctly inhibit the invasion of A549/DDP cells. Compared with that of the A549/DDP shRNA-NC+2 *μ*g/ml cisplatin group, the relative invasion rate of the A549/DDP shRNA+2 *μ*g/ml cisplatin group still decreased clearly (*F* = 0.248, *P* < 0.001). ^∗∗∗^*P* < 0.001.

**Figure 10:** RP11-838N2.3 overexpression could not affect the cell cycle of A549. (a) A549 OE-NC. (b) A549 OE. (c) A549 OE-NC+2 *μ*g/ml cisplatin. (d) A549 OE+2 *μ*g/ml cisplatin. (e) Compared with the A549 OE-NC group, the A549 OE group in the cell ratio of the G0/G1 phase (*F* = 0.578, *P* = 0.051), S phase (*F* = 0.109, *P* = 0.397), and G2/M phase (*F* = 0.649, *P* = 0.992) showed no significant difference. Under the action of cisplatin, compared with those in the A549 OE-NC+2 *μ*g/ml cisplatin group, the cell ratios in the A549 OE+2 *μ*g/ml cisplatin group in the G0/G1 phase (*F* = 6.438, *P* = 0.635), S phase (*F* = 7.866, *P* = 0.830), and G2/M phase (*F* = 0.836, *P* = 0.488) were not distinctly different.

The article "lncRNA RP11-838N2.3 Promoted Cisplatin Resistance in Lung Adenocarcinoma" was published in 2020. Journal: Biomed Res Int.

**Figure 11:** RP11-838N2.3 knockdown could not affect the cell cycle of A549/DDP. (a) A549/DDP shRNA-NC. (b) A549/DDP shRNA. (c) A549/DDP shRNA-NC+2 *μ*g/ml cisplatin. (d) A549/DDP shRNA+2 *μ*g/ml cisplatin. (e) Compared with those in the A549/DDP shRNA-NC group, the cell ratios in the A549/DDP shRNA group in the G0/G1 phase (*F* = 1.012,*P* = 0.905), S phase (*F* = 0.341, *P* = 0.221), and G2/M phase (*F* = 1.942, *P* = 0.110) were not evidently different. Under the action of cisplatin, compared with those in the A549/DDP shRNA-NC+2 *μ*g/ml cisplatin group, the cell ratios in the A549/DDP shRNA+2 *μ*g/ml cisplatin group in the G0/G1 phase (*F* = 0.958, *P* = 0.400), S phase (*F* = 11.701, *P* = 0.662), and G2/M phase (*F* = 8.507, *P* = 0.248) were not different. There were also no significant differences in the proportion of cells.

**Figure 12:** RP11-838N2.3 overexpression could affect the apoptosis of A549. (a) A549 OE-NC. (b) A549 OE. (c) A549 OE-NC+2 *μ*g/ml cisplatin. (d) A549 OE+2 *μ*g/ml cisplatin. (e) Compared with that of the A549 OE-NC group, the apoptosis rate of the A549 OE group was evidently reduced (*F* = 10.304, *P* = 0.001). Under the action of cisplatin drugs, RP11-838N2.3 overexpression still significantly inhibited the apoptosis of A549 cells. Compared with that of the A549 OE-NC+2 *μ*g/ml cisplatin group, the apoptosis rate of the A549 OE+2 *μ*g/ml cisplatin group also decreased clearly (*F* = 2.236, *P* < 0.001). ^∗∗∗^*P* < 0.001.

**Figure 13:** RP11-838N2.3 knockdown could affect the apoptosis of A549/DDP. (a) A549/DDP shRNA-NC. (b) A549/DDP shRNA. (c) A549/DDP shRNA-NC+2 *μ*g/ml cisplatin. (d) A549/DDP shRNA+2 *μ*g/ml cisplatin. (e) Compared with that of the A549/DDP shRNA-NC group, the apoptosis rate of the A549/DDP shRNA group was evidently increased (*F* = 5.828, *P* < 0.001). Under the action of cisplatin drugs, RP11-838N2.3 knockdown can also evidently promote the apoptosis of A549/DDP cells. Compared with that of the A549/DDP shRNA-NC+2 *μ*g/ml cisplatin group, the apoptosis rate of the A549/DDP shRNA+2 *μ*g/ml cisplatin group was also evidently increased (*F* = 3.322, *P* < 0.001). ^∗∗∗^*P* < 0.001.

The article "lncRNA RP11-838N2.3 Promoted Cisplatin Resistance in Lung Adenocarcinoma" was published in 2020. Journal: Biomed Res Int.

**Table 1:** Clinical features of 57 LAD patients and the relative expression levels of RP11-838N2.3.

Term	Case (*n*)	Relative expression level	Kruskal-Wallis test or Mann-Whitney *U* test	*P*
Sex			234.00	0.453
Male	28	40.21 (30.13-51.32)		
Female	29	41.42 (29.12-52.35)		
TMN stage			10.124	0.414
Ia	12	38.67 (29.54-51.56)		
Ib	28	38.92 (30.41-52.34)		
IIa	7	40.85 (30.83-51.83)		
IIb	2	41.23 (31.92-51.72)		
IIIa	8	41.10 (32.34-52.12)		
Histological degree			11.456	0.321
Poor	11	38.13 (29.12-49.23)		
Poor-moderate	7	37.43 (30.87-50.54)		
Moderate	17	40.82 (31.54-51.82)		
Moderate-high	9	41.34 (30.12-50.01)		
High	13	41.39 (31.56-51.34)		
Lymph node metastasis			3.213	0.009
Yes	14	60.37 (42.94-72.34)		
No	43	31.40 (21.84-42.84)		
Smoking			267.00	0.672
Yes	20	40.23 (30.34-51.56)		
No	37	41.56 (31.41-52.19)		

**Table 2:** Clinical characteristics between the cisplatin-sensitive group and cisplatin-insensitive group.

Term	Sensitive group (*n* = 25)	Insensitive group (*n* = 32)	*X* ^2^	*P*
Sex			0.148	0.701
Male	12	17		
Female	13	15		
TMN stage			0.686	0.953
Ia	2	1		
Ib	6	8		
IIa	7	9		
IIb	5	7		
IIIa	5	7		
Histological degree			0.338	0.987
Poor	4	5		
Poor-moderate	5	7		
Moderate	7	10		
Moderate-high	3	5		
High	5	5		
Lymph node metastasis			0.004	0.952
Yes	8	10		
No	17	22		
Smoking			0.002	0.962
Yes	10	13		
No	15	19		

## Data Availability

All datasets used in this study are included in the manuscript.
